# Deep Sentiment Analysis of Twitter Data Using a Hybrid Ghost Convolution Neural Network Model

**DOI:** 10.1155/2022/6595799

**Published:** 2022-07-18

**Authors:** Mohammed Hasan Ali Al-Abyadh, Mohamed A. M. Iesa, Hani Abdel Hafeez Abdel Azeem, Devesh Pratap Singh, Pardeep Kumar, Mohamed Abdulamir, Asadullah Jalali

**Affiliations:** ^1^College of Education in Wadi Addawasir, Prince Sattam Bin Abdulaziz University, Alkharj, Saudi Arabia; ^2^College of Education, Thamar University, Dhamar, Yemen; ^3^Umm Al Qura University, Al Qunfudah Medical College, Department of Physiology, Mecca, Saudi Arabia; ^4^Mental Health and Psychological Counseling Director of the Quality Assurance Unit, The Higher Institute of Science Administrative at Janaklis, Behera, Egypt; ^5^Department of Computer Science & Engineering Graphic Era, Deemed to Be University, Dehradun, Uttarakhand, India; ^6^FET, MRIIRS, Faridabad, India; ^7^Department of Medical Instruments Engineering Techniques, Al-Farahidi University, Baghdad 10021, Iraq; ^8^Department of Medical Instruments Engineering Techniques, Al-Turath University College, Baghdad 10021, Iraq; ^9^American University of Afghanistan, STM (Science Technology Mathematics), Kabul, Afghanistan

## Abstract

Several problems remain, despite the evident advantages of sentiment analysis of public opinion represented on Twitter and Facebook. On complicated training data, hybrid approaches may reduce sentiment mistakes. This research assesses the dependability of numerous hybrid approaches on a variety of datasets. Across domains and datasets, we compare hybrid models to singles. Text tweets and reviews are included in our deep sentiment analysis learning systems. The support vector machine (SVM), Long Short-Term Memory (LSTM), and ghost model convolution neural network (CNN) are combined to get the hybrid model. The dependability and computation time of each approach were evaluated. On all datasets, hybrid models outperform single models when deep learning and SVM are combined. The traditional models were less trustworthy, and deep learning algorithms have recently shown their enormous promise in sentiment analysis. Linear transformations are used in feature maps to eliminate duplicate or related features. The ghost unit makes ghost features by taking away attributes that are both similar and duplicated from each intrinsic feature. LSTM produces higher results but takes longer to process, while CNN needs less hyperparameter adjusting and monitoring. The effectiveness of the integrated model varies depending on the work, and all performed better than the others. For hybrid deep sentiment analysis learning models, LSTM networks, CNNs, and SVMs are needed. Hybrid models are used to compare SVM, LSTM, and CNN, and we tested each method's accuracy and errors. Deep learning-SVM hybrid models improve sentiment analysis accuracy. Experimental results have shown the accuracy of the proposed model shown 91.3 percent and 91.5 percent for datasets type 1 and 8, respectively.

## 1. Introduction

Data sentiment analysis on Twitter and Facebook is a new study area, adopting techniques built for certain data types and domains is another challenge. Deep learning algorithms have recently shown their enormous promise in sentiment analysis. It is widely used in marketing and financial forecasting, deep learning is polarised, and CNN and recurrent neural network (RNN) outperformed alternative strategies in the study. Getting close to any function, deep neural networks analyze more data more quickly and it can create a more precise quality. Deep neural networks that are computationally and parameter efficient. Each layer learns representations of the inputs [1], while certain deep learning algorithms are more dependable than others in specific industries, each has benefits and limitations. LSTM produces higher results but takes longer to process, while CNN needs less hyperparameter adjusting [2] and monitoring. The LSTM takes longer to grasp, advice combining two or more ways to get the benefits of each while avoiding technique flaws [3]. A lexicon-based sentiment analysis improvement ranging from 2% to 6%. A collaborative hybrid system may be able to defeat unified systems, the effectiveness of the integrated model varies depending on the work, and all performed better than the others. CNN, LSTM, and SVM [4] are used to analyze sentiment across domains and datasets. Data from social media, such as tweets and reviews, may also be used, the durations of tweets and reviews vary, as do the themes in each dataset. Sample sizes expressed feelings, and irrelevant data all differ. Some methodologies, such as sentiment analysis may not be applicable in other contexts. Therefore, some procedures for certain input data may be inaccurate. We investigated whether hybrid models outperformed single models regardless of dataset features. As a result, we investigate how various hybrid models perform on different datasets. In this study, we combined CNN, LSTM, and SVM, and aspects such as data and text storage in models were investigated. To begin with, the model has two potential CNN and LSTM sequences. There are presently two variants of these options: CNN with ReLU and SVM. To replicate tweets and reviews, we used word embedding. The accuracy of sentiment analysis was improved by combining models. Unlike previous activation methods, ReLU may stimulate many neurons at once. Different processes are activated. SVMs find the hyperplane that separates the two classes, and margin contains support vectors.

This study compares sentiment analysis techniques to a variety of cutting-edge methodologies. So that is all. Sections 2 and 3 discuss them, while Section 5 provides our results. Using hybrid models to increase sentiment analysis accuracy, other research techniques are described below in Section 2.

## 2. Related Work

It is simple to create hybrid models that improve picture identification by combining a CNN model with SVM. SVMs derive properties from convolutional networks, SoftMax employs the original CNN. A hybrid strategy for textual sentiment categorization and the hybrid model was evaluated on the data. Deep learning based on SVMs for classification some help with image recognition [5]. SVM or ReLU is used to classify two deep learning models, a resource-constrained deep learning system it employed CNN and SVM to classify sentiment [6]. It was put through its paces on four Hindi language datasets that examined the Internet shop evaluations using an LSTM-CNN multichannel model constructed by H-SVM. They looked through COVID-19 tweets and Facebook comments about the COVID-19 pandemic to categorize them [7]. In both studies, participants were negative, indifferent, or favourable. These models were assessed on a limited number of datasets or sample datasets. It is hard to verify and it uses BERT, a contextualized word embedding model, and FastText, a pretrained word embedding approach, to generate word vectors [8].

The algorithm was evaluated using Amazon reviews in addition to IMDb. For word embedding, we used Word2vec and BERT in our study, it recognizes tweets and reviews. CNN, LSTM, and SVM were utilized. Also employed are polarity-altering devices, sentiment lexicons, and machine learning. Many datasets have been tested. Sentiment analysis of movie reviews was used to improve a preliminary recommendation list produced by collaborative filtering and content-based approaches [9]. Tweets and reviews are social networking inputs, different datasets have different lengths, topics, and total reviews. Datasets differ in emotion and unnecessary information, sometimes sentiment analysis is erroneous or unproductive. Some input data may not be compatible with certain methods or processes. A sentiment classifier constructed from movie reviews after collaborative filtering. These studies make use of sentiment analysis and deep learning is applied to improve sentiment categorization. BERT and XLNET are two recent examples of transfer learning in sentiment analysis. BERT and XLNet are used, and these are popular NLP exercises. Both systems employ encoder/decoder networks. The transformer encoder network included six levels with two sublayers each. With attention and feed-forward sublayers, transformers can learn without repeating layers. BERT and XLNET were used to analyze sentiment and data and language testing can teach us a lot. These approaches require advanced equipment, enormous datasets, and lengthy processing periods. The parameters of BERT-Base are 110 M, whereas those of BERT-Large are 340 M and Pretraining necessitates the use of 4–16 cloud TPUs over the course of 4–16 days.

## 3. Proposed Model

This study looks at four hybrid models for sentiment analysis it necessitates the use of data, feature vectors, and hybrid algorithms. Algorithms for recognizing the polarity of emotions in a text, our research focuses on broad application models rather than difficulties. This saved us time from having to create and label new datasets for each application. A concern was avoiding privacy issues using the provided datasets, compare the sentiment analysis approaches used in the research. In other words, do the models forecast accurately regardless of the size or kind of dataset. There were eight datasets used. Review (IMDb #1 and #2, as well as Cornell): tweets from airlines, SemEval has 14,640 tweets that are either good, negative, or neutral. IMDb film, literary, and music reviews (IMDb reviews and Cornell Music Reviews). According to our findings, six of the eight datasets had almost identical sample sizes. Each dataset is either positive or negative. Priorities remain unaffected. A positive and negative coding strategy was used in this investigation. To reduce the dataset size, neutral labels were deleted, and classes have been rebalanced. K-fold cross-validation was also employed by examining all datasets. This technique eliminates bias.

### 3.1. Features of Vector Construction

The sentiment is comprised of the paper, the message, and the attributes on eight tweet and review datasets, investigated document-based sentiment analysis. Text-training data cleaning for sentiment analysis, there should be no white space, punctuation, or stop words. It replaces TF-IDF [10]. The vector was created using BERT and Word2vec. Word2vec made its debut in 2013. Unsupervised learning needs a large amount of data, Word2vec supports NxD documents and D-word embedding dimensions. Non-standard terms are not supported by Word2vec. The [UNK] symbol is used to indicate non-vocabulary words. Word2vec eliminates phrases that appear five or more times in our vocabulary databases [11]. Better results are from longer samples. They need constant input vectors and the duration of review and clarity of tweet histograms (*x*) and frequency of samples (*y*). Because we utilized many datasets, certain histograms are jagged. This might work for the models and this study compares raw data sentiment analysis algorithms.

We made use of tweets and reviews, we removed lengthy tweets and reviews, as a result, just a few samples were trimmed. Some of them do because tweets are restricted to 280 characters and databases linked to tweets are often brief. The remaining datasets range in size from 300 to 500 rows. Tthere may be a limit to the number of tweets and reviews [12]. There are various hybrid sentiment analysis models. One of the study's effective methods depicts a feature vector from a Word2vec or BERT model. Linear transformations are used in feature maps to eliminate duplicate or related features. The ghost unit makes ghost features by taking away attributes that are both similar and duplicated from each intrinsic feature. Then either CNN > LSTM or LSTM > CNN, then there's a ReLU or SVM. The ghost unit makes ghost features by taking away attributes that are both similar and duplicated from each intrinsic feature. LSTM produces higher results but takes longer to process, while CNN needs less hyperparameter adjusting and monitoring.

### 3.2. Emotional Analysis

When these two variants are combined, four hybrid approaches are produced: W2V/BERT vs. CNN vs. LSTM vs. SVM. We created feature vectors in two ways, all words in our training datasets were included using Word2vec. It is incapable of handling complex semantic or polymorphic scenarios; the tweets and reviews were used to make feature vectors that hybrid models could use to classify. The CNN and LSTM deep learning models are then combined to enhance sentiment analysis [13–16]. CNN processes and transmits information from one layer to the next, convolutional, and pooling/subsampling layers are combined in this layer. This study makes use of a single directional CNN and RNN input, output, and a memory cell are all part of the LSTM block. RNNs, unlike CNNs, thrive on temporal cues. Unlike LSTM, multilayer CNN may learn local information; therefore, it blends the best of both the proposed model worlds. RNN forget, input and output are all LSTM gates, these are near input, output, and memory blocks. RNNs analyze geographical data better than temporal signals, CNNs and LSTMs can learn local data, this combines space and time.

Figure 1 depicts the proposed model, which takes datasets and processes them with Word2vec before transferring the features to the ghost CNN model and LSTM in parallel. The processes generated by the ghost CNN model are sent to LSTM, which is then followed by fully connected layers. It is then processed with ReLu and SVm to generate output. The feature vectors obtained from the second layer of LSTM are transferred to the ghost CNN model, which is followed by fully connected layers and then SVM and ReLu to create output. The output of both layers is integrated to provide an accurate result. Because of the high convergence, ReLU activates function rather than Sigmoid in high-dimensional NLP. The SVM algorithm is a classification algorithm that has been used previously. We employed linear SVMs for categorising in our study, while SVM was chosen for classification because of its NLP performance. SVMs can classify and predict and its extensive use has helped many regions using linear SVMs and hybrid deep learning models, we categorised the data, the top hidden layer feature vectors were predicted using SVM. The top hidden layer feature vectors were predicted using SVM, and the Hybrid ghost model [17, 18] CNN-LSTM-SVM, the design of the hybrid model further information is provided below.

**Scenario 1 .**

Hybrid LSTM-CNN

First, consider an LSTM-CNN hybrid.  Table 1 the accuracy of the proposed model and traditional models with word2vec and BERT for 8 types of datasets. Filters of 512, 256, and 128 bits and three kernels are available. The classifier receives a 1500 matrix from the LSTM layer. It has two layers that each have 128 nodes and an output layer that is activated by the ReLU method, which is used to make it work.

**Scenario 2 .**

Hybrid LSTM-CNN Models

Preprocessing is the process of transforming data in preparation for embedding [19–23]. LSTM is the first layer, the hybrid deep learning model requires a matrix of 13, 500 following that, we have CNN. Three convolution layers receive and analyze the input. It is effective and classifies using an output layer with a ReLU activation function and two layers of 128 nodes each. As a result, the classifier was removed in this scenario, but the deep learning steps were employed. SVM is a classifier that may be used in lieu of CNN-based ReLU. Scenario 1 makes use of CNN-LSTM, whereas Situation 2 makes use of LSTM-CNN.

## 4. Experimental Outcome

We investigate deep learning (SVM, CNN, and LSTM), and a total of one preprocessed text data set was evaluated. The accuracy, F-score, adjusted rand index, statistical similarity, and completeness of the models were examined. Prior to testing, the settings, hardware devices, and library capabilities were configured. Reviews received 4 echoes, while tweets received 128. The most used K-fold validation numbers are 10, 5, and 3, significant subsets may be supported if the dataset is big enough. The k-fold cross-validation configuration option lets users determine the number of dataset folds, *k* = 10 is the most common number for assessing models in applied machine learning, but *k* = 3, *k* = 5, and *k* = 10 are all common. The datasets used in this investigation are provided below. Each validation has nine sections for training and one for testing. *k* is selected to ensure that each sample accurately represents the dataset. All cross-validation models use the same sized training sets, to compare model performance, it is ideal to divide the data into equal samples. According to a proposed model, 1,161 tweets (22.5 percent) and 1,246 retweets were generated. The proposed model had 13.3 percent (13.6 percentage points) of the same number of postings as humans, but they had more on the first level.

An illustration of this is the magnitude of the first and second level communication, the second level of communication follows the first. Using the proposed model score of 3.5 as a baseline, human-produced material outnumbers the proposed model-produced content in secondary communication. The proposed model spreads 121 items on the first and second tiers shown in Figure 2. The horizontal axis reflects the proportion of the 121 stories that include the proposed model content, while the vertical axis shows the same percentage. The retweet histogram is located slightly to the left of the tweeting histogram. The proposed model is more common among those who disseminate first-level articles. The proposed model may provide up to 70% of dissemination for some publications, although, for the most part, the proposed model provides 10% to 50%. The proposed model contributes to general retweets less than 35% of the time and first-level diffusion are significantly connected.

Figure 3 depicts communication on both the main and secondary levels, with some users scoring higher than 0, but more users scoring lower than 0. The suggested model score distribution is notably biassed to the right, with the most concentrated distribution of users scoring below 0.2. The suggested model scores of the most popular users are clearly biassed to the right, with scores concentrating between [0, 0.15], a far higher concentration than the entire user sample. Most active users had a wider dispersion in the high-proposed model score interval than the entire sample and high-impact users. Regular tweeters are included in the proposed model, although they are not important persons who receive many retweets.

Figure 4 depicts human users' responses and conditional probability distribution score vs. rate of the proposed model-initiated retweets. The lighter line indicates that when the tweeter is a proposed model, humans do the bulk of retweets. Most people prefer to retweet news from human users rather than news from major distributors in the proposed model. The results of applying sentiment-based dimension reduction to the Twitter dataset are shown in Table 2 and Figure 5.

Table 1 shows the accuracy of the proposed model convolution neural network, support vector machine, long short-term memory, proposed model without LSTM, proposed model without CNN, proposed model without SVM, and LSTM without SVM. The accuracy of the proposed model is better than other models in almost all datasets.

### 4.1. The Proposed Hybrid Methods' Outcomes are Compared to the Baseline Procedures

We ran Word2vec and a pre-trained BERT model through their paces twice, in the proposed model situations, a pre-trained BERT model achieves more than 90% accuracy. Seven of the eight datasets were hybrid in nature (SVM, CNN, or LSTM) [24–27].  Table 1 displays the proposed model's accuracy statistics for music and book reviews. Results were better when the CNN-SVM model was used. It boosted them by 91.3 percent and 91.5 for datasets type 1 and 8, respectively. The hybrid model outperformed solo deep learning models in terms of F-score. The AUC of hybrid and solo deep learning models is compared with hybrid SVM models, 6/8 Word2vec datasets fared better. Tweets Airline and IMDb movie reviews have the highest overall ratings. These strategies are effective for evaluating books and music. The sentiment 140 dataset is erroneous and several data samples of varying lengths are used.

The pre-trained BERT outperforms Word2vec for sentiment analysis. Hybrid models, on the other hand, outperform other models for each dataset. Word2vec and BERT models were outperformed by hybrid models. Pretrained BERT for sentiment analysis is better than Word2vec for all models and datasets, hybrid models perform well for every dataset we analyze. Word2vec and BERT alone failed, single Word2vec models are inaccurate. Despite these models' 90% accuracy, BERT has improved outcomes. Hybrid Word2Vec models outperform single model because of their great precision, the results using BERT have also gotten better, but only a little (usually more than 90%). For lengthier texts, LCNN-SVN beats other hybrid models, the length of the reviews ranges from 1 to 800 words. It is a shame that Cornell's film assessments are not more widely circulated. The sample length distribution in the Sentiment140 dataset is skewed. Sentiment140 and Cornell film reviews performed worse than the others; similarly, make use of a single tweet or review dataset and hybrid model boost processing speed and accuracy.

Algorithmic performance, as well as model dependability, are critical; other options include layer count, input matrix size, and other algorithm-dependent characteristics. CNN examines the convolution kernels and output channels of each layer and the root mean square error is low as shown in Figure 6. In practice, hybrid vehicles' enhanced dependability comes at a cost. Maximum network layers are defined by model design, activation function, optimization strategy, and other considerations. ResNets can handle up to a thousand layers for CIFAR-10, as you said. Kaiming initialization kept the variance of each layer's activations at roughly 1, while Xavier initialization is better for sigmoid activation functions. As ReLU functions gained prominence, Kaiming initialization grew increasingly prevalent. As ReLU functions gained prominence, Kaiming initialization enabled deeper network training. We look at the time it takes to make a model in the comparison analysis because it shows how complicated it is to run. It takes time to train and evaluate the Word2vec and BERT models. It simply divides the data and configures the categorization model (number of layers and nodes per layer). Hybrid models that use BERT for feature extraction are often more accurate than Word2vec, although they take longer to process. Deep learning on a regular basis beats hybrid technique. They frequently outperform across datasets; emotion categorization necessitates feature extraction. For feature extraction, investigated TF-IDF and word embedding. Shorter processing times result in greater and more consistent results. Due to their complexity and parameterization, hybrid models take longer to compute than single models. Feature extraction using TF-IDF and word embedding, processing time increases. Since hybrid models are more sophisticated and contain more parameters, they take longer to process. Processing time may be compared to accuracy, even with long computations. The proposed hybrid deep learning model works on various data sets, the goal of this model is to create a cross-domain hybrid deep learning model for sentiment analysis. It may be appropriate for certain datasets but not for others, owing to the need to determine multiple parameters. Previous experiments yielded the following results: they took longer to compute, but they outperformed single models on all datasets. In combination with CNN, LSTM, and SVM, SVM can categorize and store previous data at state nodes (cell states). SVM enhanced the outcomes of L-CNN and C-LSTM.

## 5. Conclusion

To analyze social network sentiment, we suggest using hybrid deep learning models. Our datasets included eight tweet and review datasets, and then we compared four hybrid automobiles to a single hybrid vehicle. The purpose of this research is to evaluate the adaptability of hybrid models to a broad variety of dataset kinds and sizes. There is a strong connection between the quality of the data and the reliability of sentiment polarity analysis. All the other models we tried failed to analyze sentiment polarity. For sentiment analysis, combining deep learning and SVM models beats utilizing standalone models. In most circumstances, SVM hybrid models outperform non-SVM hybrid models in terms of dependability, although they require a much longer time to calculate. The quality of the datasets has a significant impact on the algorithms' performance. To understand more about business, marketing, and medicine, a range of hybrid datasets and settings are required. Its goal is to offer people comprehensive personal input. Several problems remain, despite the evident advantages of sentiment analysis of public opinion represented on Twitter and Facebook. On complicated training data, hybrid approaches may reduce sentiment mistakes. This research assesses the dependability of numerous hybrid approaches on a variety of datasets. Across domains and datasets, we compare hybrid models to singles. Text tweets and reviews may be included in our deep sentiment analysis learning systems. The SVM, LSTM, and ghost CNN models are compared. The dependability and computation time of each approach were evaluated. On all datasets, hybrid models outperform single models when deep learning and SVM are combined. The proposed model was less trustworthy. We wish to try hybrid approaches for sentiment analysis on hybrid datasets and hybrid settings to better understand business, marketing, or health. This helps us comprehend the field. It uses sentiment analysis and contextual association to personalise comments and recommendations.

## Figures and Tables

**Figure 1:** The proposed model.

**Figure 2:** First and second level communication get a 0-1 user contribution score.

**Figure 3:** Primary and secondary communication by the proposed model.

**Figure 4:** Conditional probability distribution of the proposed model scores of the proposed model sides of the forwarding relationship.

**Figure 5:** Comparison of the proposed model with the SVM based model.

**Figure 6:** The number of convolution kernels RMSE fluctuation.

**Table 1:** The accuracy of the proposed model and traditional models with Word2vec and BERT for 8 types of datasets.

Datasets	CNN	SVM	LSTM	Proposed model-LSTM	Proposed model-CNN	Proposed model-SVM	LSTM-SVM	Proposed model
1	85.3	89.8	80.4	80.2	89.9	**80.7**	89.9	91.3
2	83.3	87.8	88.2	88.0	88.6	**88.7**	88.8	89.4
3	80.6	85.5	**87.5**	86.0	87.3	86.7	86.8	87.9
4	88.9	88.7	88.6	89.8	90.0	90.0	**90.4**	90.6
5	83.8	88.4	86.2	89.3	**89.5**	**89.5**	**89.5**	89.4
6	78.8	83.5	87.2	84.0	**87.5**	87.3	86.9	87.6
7	88.3	87.5	88.3	86.8	84.6	88.8	**84.8**	88.9
8	87.7	87.6	89.7	80.9	83.2	87.7	**83.8**	91.5

**Table 2:** Demonstrates how the suggested method improves opinion text grouping and results.

Methods	Accurateness	*F*-score	Adjusted rand index	Statistical similarity	Completeness
DeepCoNN-BERT	0.62	0.606	0.0388	0.0326	0.0328
ConvMF	0.598	0.595	0.0388	0.0325	0.0327
SVM	0.607	0.602	0.0378	0.0308	0.0320
SVM + LSTM	0.624	0.609	0.0387	0.0332	0.0335
Proposed model	0.648	0.647	0.2470	0.2020	0.2020

## Data Availability

The dataset has been collected through tweepy library using Python.
